The article "Sulodexide Prevents Peritoneal Fibrosis by Downregulating the Expression of TGF-β1 and Its Signaling Pathway Molecules" was retracted in 2023. Reasons: signs of a paper mill; compromised peer review; unreliable results or conclusions.

# Sulodexide Prevents Peritoneal Fibrosis by Downregulating the Expression of TGF-*β*1 and Its Signaling Pathway Molecules

**DOI:** 10.1155/2021/2052787

**Published:** 2021-08-30

**Authors:** Zhiqiang Duan, Jia Yao, Nan Duan, Min Wang, Shiwei Wang

**Affiliations:** ^**1**^ Department of Renal Disease, People's Hospital of Tang County (The Fourth Central Hospital of Baoding City), Baoding, Hebei 072350, China; ^**2**^ Department of Geriatrics, Traditional Chinese Medicine Hospital of Wangdu County, Baoding, Hebei 072450, China

## Abstract

Peritoneal dialysis is one of the main renal replacement treatments. However, long-term peritoneal dialysis keeps the peritoneum in contact with the sugar-containing nonphysiological peritoneal fluid, which leads to recurrent peritonitis, peritoneal fibrosis, and failure of ultrafiltration. Transforming growth factor-*β*1 (TGF-*β*1), related cytokines, and inflammatory factors are closely related to peritoneal fibrosis. Sulodexide (SLX) is a new type of glycosaminoglycan preparation, which is involved in the formation of an anionic charge barrier and can maintain the selective permeability of vascular endothelial cells. In this study, the innovative analysis of SLX specifically prevents the process of peritoneal dialysis peritoneal fibrosis by downregulating the expression of TGF-*β*1 and its signaling pathway molecules. We randomly divided 30 rats into three groups. The blank control group received no treatment. The peritoneal dialysis model group was injected with 4.25% peritoneal dialysate (PDF) 20 ml daily, and the SLX group was injected with 4.25% PDF 20 ml + sulodexide (SLX) 20 mg/kg daily. After 8 weeks of dialysis, the rats were sacrificed, and the peritoneal function test was performed to determine the amount of glucose transport and ultrafiltration. The thickness of peritoneal per unit area was observed under high magnification. The level of inflammation in peritoneal tissue and the expression of TGF-*β*1/Smad were detected. The results showed that SLX can significantly improve peritoneal tissue thickening and inflammation, can downregulate the expression of TGF-*β*1, Smad2, Smad3, and Smad7 in peritoneal tissue, and improve the progression of peritoneal fibrosis.

## 1. Introduction

Peritoneal dialysis is one of the main alternative treatments for patients with end-stage renal disease. It can delay the decline of residual renal function, provide continuous filtration, has a good removal effect on middle molecular toxins, and helps in blood pressure and body fluid balance [1–3]. However, long-term peritoneal dialysis keeps the peritoneum in contact with the sugar-containing nonphysiological peritoneal dialysis fluid, causing repeated episodes of peritonitis, which can lead to peritoneal fibrosis, resulting in the failure of ultrafiltration, and finally leading to the withdrawal of patients from peritoneal dialysis treatment, which significantly limits the development of peritoneal dialysis. Long-term exposure of the patient's peritoneum to biocompatible dialysate with high blood glucose concentration and peritonitis caused by operation can also impair peritoneal function [4, 5]. In addition, some patients develop encapsulating peritoneal sclerosis, which is a rare excessive peritoneal fibrosis with high mortality [6]. So far, there has been no specific and effective therapy that can be used to prevent or inhibit the process of peritoneal fibrosis.

The article "Sulodexide Prevents Peritoneal Fibrosis by Downregulating the Expression of TGF-β1 and Its Signaling Pathway Molecules" was retracted in 2023. Reasons: signs of a paper mill; compromised peer review; unreliable results or conclusions.

Clinical studies have shown that transforming growth factor-*β*1 (TGF-*β*1), related cytokines, and inflammatory factors are closely related to peritoneal fibrosis. TGF-*β*1 is considered to be the most critical cytokine in the pathogenesis of peritoneal fibrosis, which can regulate cell proliferation and differentiation, promote the formation of an extracellular matrix, participate in the regulation of embryonic development, etc., mainly through the activation of its downstream signal protein Smads [7–11]. Other studies have shown that in various acute and chronic inflammatory states, peritoneal mesothelial cells are damaged, and macrophages are activated to participate in the formation of peritoneal fibrosis by secreting a large number of inflammatory cytokines, growth factors, matrix proteins, etc. [12]. Studies have also shown that high glucose conditions in dialysate and inflammatory factors can increase the expression of TGF-*β* [13]. TGF-*β* induces the connective tissue growth factor (CTGF), which is the main factor controlling fibrosis in all organs. Therefore, the current prevention and treatment of peritoneal fibrosis is mainly aimed at promoting fibrotic cytokines such as TGF-*β*1.

Sulodexide (SLX) is a new type of glycosaminoglycan preparation that has a strong antithrombotic effect on arteries and veins. It participates in the formation of an anionic charge barrier and can also maintain the selective permeability of vascular endothelial cells [14]. The pharmacological effects of SLX also include maintaining vascular wall permeability selectivity by preserving normal negative charges in the vascular wall and inhibiting cell proliferation and subsequent loss of vascular wall basement membrane and extracellular matrix function. The selective effect of SLX in maintaining vascular wall permeability can prevent the common transvascular leakage of different macromolecules (such as albumin, fibrinogen, and lipoprotein). The leakage of these macromolecules is an early symptom of atherosclerosis, manifested in kidney disease as proteinuria. Studies have shown that SLX regulates cell proliferation and adhesion by binding and isolating TGF-*β*1, can regulate peritoneal inflammation, and is also involved in the process of damage repair and fibrosis [15]. Therefore, this study innovatively analyzed the effect of SLX on the peritoneal tissue inflammation and the expression of TGF-*β*1 and its signaling pathway molecules in peritoneal dialysis model rats and explored the application value of SLX in preventing peritoneal dialysis and peritoneal fibrosis, in order to provide more experimental data and program references for peritoneal dialysis treatment.

The article "Sulodexide Prevents Peritoneal Fibrosis by Downregulating the Expression of TGF-β1 and Its Signaling Pathway Molecules" was retracted in 2023. Reasons: signs of a paper mill; compromised peer review; unreliable results or conclusions.

## 2. Materials and Methods

### 2.1. Animal Source

Thirty SPF SD rats, 8–10 weeks old, half female and half male, weighing 180–250 g, were purchased from Shanghai Slack Laboratory Animal Co., Ltd, Animal production license number: SCXK (Shanghai) 2017–0005. Rats were housed in rodent cages in room 22, which has a 12-hour light-dark cycle, and standard rat food and water were given.

### 2.2. Specific Method

#### 2.2.1. Animal Modeling and Grouping

Thirty rats were randomly divided into three groups: blank control group, peritoneal dialysis model group, and SLX group. The blank control group did not receive any treatment [16]. In the peritoneal dialysis model group and SLX group a self-made peritoneal dialysis tube was inserted into the abdominal cavity, and peritoneal dialysis was performed once a day for 8 weeks to complete the rat model. In the peritoneal dialysis model group, 20 ml of 4.25% peritoneal dialysate (PDS) was injected at the same time every day, and the SLX group was injected with 4.25% PDS 20 ml + SLX 20 mg/kg at the same time every day.

#### 2.2.2. Peritoneal Function Test

After the end of the dosing cycle, the rats were intraperitoneally injected with 4.25% dianeal peritoneal dialysate (lactate-G 4.25%). After 4 hours, the rats were anesthetized to open the peritoneum and take out the fluid for ultrafiltration volume determination (ultrafiltration volume = the amount of liquid taken out after 4 h − the amount of fluid given). 2 ml of rat tail vein blood was drawn at 0 and 4h, respectively, and the glucose concentration was measured by the automatic biochemical analyzer, and the glucose transport volume was calculated. Formula: glucose transport volume mmol·kg^−1^ = (initial glucose concentration × injected into dialysate volume) − (glucose concentration at the end × dialysate volume at the end).

#### 2.2.3. Measurement of Peritoneal Thickness

The rats were sacrificed, and peritoneal samples were collected and fixed in 10% formaldehyde buffer solution to make 3 *μ*m thick sections. Pathological staining was performed. The full length of the peritoneum was measured using a microscope at 400 times magnification, and the thickness of the peritoneum was measured at 3 different positions in each field of view, and the average value was taken. The results were displayed in the form of a statistical graph.

The article "Sulodexide Prevents Peritoneal Fibrosis by Downregulating the Expression of TGF-β1 and Its Signaling Pathway Molecules" was retracted in 2023. Reasons: signs of a paper mill; compromised peer review; unreliable results or conclusions.

#### 2.2.4. Detection of Inflammation Levels

Enzyme-linked immunosorbent assay (ELISA) was used to detect the expression levels of interleukin-1*β* (IL-1*β*), tumor necrosis factor-*α* (TNF-*α*), and interleukin-6 (IL-6) in peritoneal tissues. IL-1*β*, TNF-*α*, IL-6 related ELISA kits were purchased from Shanghai Enzyme Link Biotechnology Co., Ltd. The peritoneal tissue was washed and cut into small pieces and put into a beaker. After the homogenate was added, it was thoroughly ground by a homogenizer. After the homogenate was added again, it was centrifuged at 43,000 r/min for 30 minutes, and the supernatant was taken for use. After room temperature equilibration, the supernatant was sequentially added to the blank control wells of the test plate and the standard wells of the sample wells, and horseradish peroxidase-labeled antibodies were sequentially added for incubation. The plates were washed sequentially, and the substrate was added. After the reaction is complete, the stop solution is added to stop the reaction. The absorbance of each well at 450 nm was detected, and the expression levels of IL-1*β*, TNF-*α*, and IL-6 were calculated according to the equation after a standard curve was drawn.

#### 2.2.5. Analysis of the Expression of TGF-*β*1/Smad

QRT-PCR was used to detect the expression of TGF-*β*1/Smad in peritoneal tissues. 1g of the peritoneal sample was taken out, RNAiso Plus kit (Thermo Fisher) was used to extract the total RNA from peritoneal tissue, reverse transcription kit (Thermo Fisher) was used for cDNA synthesis, and SYBR Green I Master Mix kit (Thermo Fisher) was used for the reaction on a real-time fluorescence quantitative PCR machine (Thermo Fisher) with GAPDH as the internal reference gene. The primer design was shown in Table 1. The relative expression levels of TGF-*β*1, Smad2, Smad3, and Smad7 were calculated according to the 2^−ΔΔCt^ method [17]. Reaction system (25 *μ*l): 2 *μ*l cDNA, 12.5 *μ*l SYBR Green I Master Mix, 1 *μ*l forward primer, 1 *μ*l reverse primer, 8.5 *μ*l DEPC water. The reaction parameters: 95°C for 20s; then 95°C for 10s, 70°C for 20s, 60°C for 15s, 35 cycles.

### 2.3. Statistical Method

SPSS21.0 software was used for statistical analysis, and GraghPad prism 8 was used for statistical mapping. The measurement data were expressed as mean ± standard deviation, the comparison between groups was performed by the Student's *t*-test, and the one-way analysis of variance was used for comparison. *P* < 0.05 indicates that the difference is statistically significant.

The article "Sulodexide Prevents Peritoneal Fibrosis by Downregulating the Expression of TGF-β1 and Its Signaling Pathway Molecules" was retracted in 2023. Reasons: signs of a paper mill; compromised peer review; unreliable results or conclusions.

## 3. Results

### 3.1. Changes in Glucose Transport Volume, Ultrafiltration Volume, and Peritoneal Thickness in Peritoneal Dialysis Rats

To explore the effects of peritoneal dialysis on rats, we compared the changes in glucose transport, ultrafiltration, and peritoneal thickness in the blank control group and the peritoneal dialysis model group. The results showed that compared with the blank control group, the glucose transport volume and peritoneal thickness of the peritoneal dialysis model group were increased, and the ultrafiltration volume level was significantly reduced, and the difference was statistically significant (*P* > 0.05), as shown in Figure 1.

### 3.2. Inflammatory Progression of Peritoneal Tissue in Peritoneal Dialysis Rats

To analyze the inflammatory progress of peritoneal dialysis on rat peritoneal tissues, we extracted the peritoneal tissues of the blank control group and peritoneal dialysis model group for tissue homogenization to detect the expression of inflammatory factors. The results showed that compared with the blank control group, the levels of IL-*β*, TNF-*α*, and IL-6 in the peritoneal tissue of the peritoneal dialysis model group were significantly increased, and the differences were statistically significant (*P* > 0.05), as shown in Figure 2.

### 3.3. Expression of TGF-*β*1/Smad in Peritoneal Tissue of Peritoneal Dialysis Rats

To study the expression of TGF-*β*1/Smad in rat peritoneal tissues after peritoneal dialysis, we detected TGF-*β*1/Smad mRNA in peritoneal tissues of the blank control group and peritoneal dialysis model group. The results showed that compared with the blank control group, the levels of TGF-*β*1, Smad2, Smad3, and Smad7 in the peritoneal tissue of the peritoneal dialysis model group were significantly increased, and the differences were statistically significant (*P* > 0.01), as shown in Figure 3.

### 3.4. The Effect of SLX on Improving Glucose Transport Volume, Ultrafiltration Volume, and Peritoneal Tissue Thickness in Peritoneal Dialysis Rats

To explore the effects of SLX on peritoneal dialysis rats, we compared the changes in glucose transport, ultrafiltration, and peritoneal thickness between the peritoneal dialysis model group and the SLX group. The results showed that compared with the rats in the peritoneal dialysis model group, the SLX group rats had lower glucose transport volume, peritoneal thickness, and significantly higher levels of ultrafiltration, and the differences were statistically significant (*P* > 0.05), as shown in Figure 4.

The article "Sulodexide Prevents Peritoneal Fibrosis by Downregulating the Expression of TGF-β1 and Its Signaling Pathway Molecules" was retracted in 2023. Reasons: signs of a paper mill; compromised peer review; unreliable results or conclusions.

### 3.5. SLX Can Inhibit the Inflammatory Progression of Peritoneal Tissue in Peritoneal Dialysis Rats

In order to explore the inflammatory progress of SLX on the peritoneal tissue of peritoneal dialysis rats, we extracted the peritoneal tissues of the peritoneal dialysis model group and the SLX group for tissue homogenization to detect the expression of inflammatory factors. The results showed that compared with rats in the peritoneal dialysis model group, the levels of IL-*β*, TNF-*α*, and IL-6 in the peritoneal tissue of the SLX group were significantly reduced, and the differences were statistically significant (*P* > 0.05), as shown in Figure 5.

### 3.6. SLX Can Reduce the Expression of TGF-*β*1/Smad in Peritoneal Tissues of Peritoneal Dialysis Rats

To study the effect of SLX on the expression of TGF-*β*1/Smad in rat peritoneal tissues after peritoneal dialysis, we detected TGF-*β*1/Smad mRNA in peritoneal tissues of rats in the peritoneal dialysis model group and SLX group. The results showed that compared with rats in the peritoneal dialysis model group, the levels of TGF-*β*1, Smad2, Smad3, and Smad7 in the peritoneal tissues of the SLX group were significantly reduced, and the differences were statistically significant (*P* > 0.01), as shown in Figure 6.

## 4. Discussion

Peritoneal dialysis uses the peritoneum as a semipermeable membrane to regularly infuse the prepared dialysate into the patient's peritoneal cavity through the action of gravity [18]. The peritoneal dialysate is constantly replaced to achieve the purpose of removing metabolites and toxic substances in the body and correcting the disorder of water and electrolyte balance. Although peritoneal dialysis is a good treatment method for clearing the molecular toxins in the body of patients with acute kidney injury and chronic renal failure, its improper operation, incision and tube infection, patient immunity, dialysate contamination, and advanced age can cause a series of complications [19, 20]. Among them, peritoneal fibrosis is one of the most serious complications in patients undergoing continuous ambulatory peritoneal dialysis and is the main cause of interruption of peritoneal dialysis treatment. The high concentration of glucose in the peritoneal dialysis fluid is a key driver of peritoneal dialysis and is considered to be an important initial factor in the development of peritoneal fibrosis. Long-term exposure to peritoneal dialysis is related to the development of peritoneal function and structural changes. The changes observed after peritoneal dialysis are mesothelial shedding, mesenchymal transformation of peritoneal mesothelial cells, submesothelial extracellular matrix deposition, and fibrosis [21]. In this study, SD rats were treated with peritoneal dialysis, and it was observed that compared with the blank control group, the glucose transport volume and peritoneal thickness of the peritoneal dialysis model group were increased, and the ultrafiltration volume level was significantly reduced. It suggests that the changes caused by peritoneal dialysis will lead to changes in peritoneal morphology and function, increase in glucose transport, and ultimately lead to the failure of ultrafiltration.

The article "Sulodexide Prevents Peritoneal Fibrosis by Downregulating the Expression of TGF-β1 and Its Signaling Pathway Molecules" was retracted in 2023. Reasons: signs of a paper mill; compromised peer review; unreliable results or conclusions.

A variety of profibrotic cytokines are closely related to peritoneal fibrosis. TGF-*β*1 is a key molecule in the process of fibrosis in a variety of tissues and organs, including peritoneal tissue, and it plays a role mainly through the phosphorylation of its signaling pathway protein Smad [22]. TGF-*β*1 is also a multifunctional inflammatory factor [23]. Studies have shown that long-term stimulation of inflammatory factors can lead to the transdifferentiation of peritoneal mesothelial cells to myofibroblasts, which is also the early stage of fibrosis of peritoneal mesothelial cells [24]. In our study, we analyzed the inflammatory progression of rat peritoneal tissue and the expression of TGF-*β*1/Smad by peritoneal dialysis. Compared with the blank control group, the peritoneal tissue inflammatory factors, IL-*β* and TNF, in the peritoneal dialysis model group were compared. The levels of *α* and IL-6 increased significantly, and the levels of TGF-*β*1, Smad2, Smad3, and Smad7 in the peritoneal tissue of rats increased significantly. This result is consistent with the above theory, suggesting that peritoneal dialysis can promote the inflammatory progression of peritoneal tissue and may be regulated by the expression of TGF-*β*1/Smad. Therefore, the TGF-*β*1/Smad pathway may become a therapeutic target that affects the progression of peritoneal fibrosis.

Studies have found that the connection between peritoneal mesothelial cells can change the structure and function of the peritoneum [25]. Under normal circumstances, the surface of peritoneal mesothelial cells is surrounded by a mechanical defense barrier, which is composed of glycosaminoglycans, proteoglycans, and phospholipids, which can form a smooth, nonadhesive serosal layer to protect the peritoneum from abrasion, infection, and tumor spread. Glycosaminoglycans include heparan sulfate, chondroitin sulfate, keratan sulfate, hyaluronic acid, etc.; proteoglycans are mainly synthesized by decorin and disaccharides. It has been reported in foreign literature that human peritoneal mesodermal cells can synthesize and secrete proteoglycan, dioglycan, basement membrane polysaccharide, and hyaluronic acid in vitro studies, and hyaluronic acid, proteoglycan and dioglycan were simultaneously found in peritoneal dialysate [26]. SLX is a new glycosaminoglycan preparation, currently clinically, which is mainly composed of 80% heparan sulfate and 20% dermatan sulfate in electrophoresis. SLX not only has the effects of anticoagulation, thrombolysis, anticardiovascular disease, lowering blood lipids, etc. but also has unique effects in the treatment of diabetic nephropathy: protecting and rebuilding the vascular endothelium of vascular damage, maintaining the charge barrier of the glomerular basement membrane, reducing albumin permeability, and other protective effects on the kidneys [27]. Therefore, we believe that exogenous supplementation of SLX has a protective effect on the peritoneum.

The article "Sulodexide Prevents Peritoneal Fibrosis by Downregulating the Expression of TGF-β1 and Its Signaling Pathway Molecules" was retracted in 2023. Reasons: signs of a paper mill; compromised peer review; unreliable results or conclusions.

Therefore, in order to explore the effect of SLX on the peritoneal tissue of peritoneal dialysis rats, we injected SLX into the peritoneal cavity of peritoneal dialysis model rats, and extracted the peritoneal tissue of rats in the SLX group for tissue homogenization. The test results found that compared with rats in the peritoneal dialysis model group, rats in the SLX group had decreased glucose transport and peritoneal thickness, and significantly increased the level of ultrafiltration. It is suggested that SLX has a protective effect on peritoneal tissue and can reduce the damage caused by peritoneal dialysis. We explored the inflammatory progression of SLX on the peritoneal tissue of peritoneal dialysis rats and found that the levels of IL-*β*, TNF-*α*, and IL-6 in the peritoneal tissue of rats in the SLX group were significantly reduced, and the levels of TGF-*β*1, Smad2, Smad3, and Smad7 were also significantly reduced. It is suggested that SLX can reduce the inflammatory level in peritoneal tissues and downregulate the expression of TGF-*β*1/Smad. The reason may be that the exogenous addition of SLX can inhibit the increase of the inflammatory factors and TGF-*β*1/Smad induced by peritoneal dialysate. Under the action of peritoneal dialysate, the protein content of hyaluronic acid and proteoglycan in peritoneal mesothelial cells increases [28]. We believe that the increase in the expression of hyaluronic acid and proteoglycan may be a self-protective response of the cell, and it increases with the stimulation time; the mechanical defense barrier on the peritoneal surface gradually consumes damage, and the expression of hyaluronic acid and proteoglycan protein gradually decreases. Moreover, the increased reactivity of hyaluronic acid and proteoglycan is insufficient to protect the peritoneum, so the expression of inflammatory factors and TGF-*β*1/Smad increases. After the supplementation of exogenous SLX, the content of hyaluronic acid and proteoglycan protein increased significantly. Therefore, the supplementation of SLX repaired the mechanical defense barrier and protected the peritoneal function, and the expression of TGF-*β*1/Smad decreased gradually.

The article "Sulodexide Prevents Peritoneal Fibrosis by Downregulating the Expression of TGF-β1 and Its Signaling Pathway Molecules" was retracted in 2023. Reasons: signs of a paper mill; compromised peer review; unreliable results or conclusions.

To sum up, SLX can significantly improve peritoneal tissue thickening and inflammation, downregulate the expression of TGF-*β*1, Smad2, Smad3, and Smad7 in peritoneal tissue, and improve the progress of peritoneal fibrosis. This study can provide an experimental theoretical basis for the treatment of peritoneal fibrosis in clinical peritoneal dialysis patients, and subsequent clinical trials can be conducted appropriately to explore the safety of the drug.

## Figures and Tables

**Figure 1:** Changes in glucose transport volume, ultrafiltration volume, and peritoneal thickness in peritoneal dialysis rats. (a) Glucose transport volume, (b) ultrafiltration volume, and (c) peritoneal thickness; compared with the blank control group, ^*∗*^*P* < 0.05.

**Figure 2:** Inflammatory progression of peritoneal tissue in peritoneal dialysis rats. The levels of inflammatory factors IL-*β*, TNF-*α*, and IL-6; compared with the blank control group, ^*∗*^*P* < 0.05.

**Figure 3:** The expression of TGF-*β*1/Smad in the peritoneal tissue of peritoneal dialysis rats. (a) TGF-*β*1 mRNA expression; (b) Smad2, Smad3, and Smad7 mRNA expression; compared with the blank control group, ^*∗∗*^*P* < 0.01.

**Figure 4:** The effect of SLX on improving the glucose transport volume, ultrafiltration volume, and peritoneal tissue thickness in peritoneal dialysis rats. (a) Glucose transport volume, (b) ultrafiltration volume, and (c) peritoneal thickness; compared with the peritoneal dialysis model group, ^*∗*^*P* < 0.05.

**Figure 5:** SLX can inhibit the inflammatory progression of peritoneal tissue in peritoneal dialysis rats. The levels of inflammatory factors IL-*β*, TNF-*α*, and IL-6; compared with the blank control group, ^*∗*^*P* < 0.05.

**Figure 6:** SLX can reduce the expression of TGF-*β*1/Smad in peritoneal tissues of peritoneal dialysis rats. (a) TGF-*β*1 mRNA expression and (b) Smad2, Smad3, and Smad7 mRNA expression; compared with the blank control group, ^*∗∗*^*P* < 0.01.

**Table 1:** Related primer sequence.

Primer sequence	Forward (5′—3′)	Reverse (5′—3′)
TGF-*β*1	TGGAAATCAATGGGATCAGTC	GAGCAAGTGCTTGGTATGG
Smad2	AGGACGATTAGATGAGCTTGAG	GAGCAAGTGCTTGGTATGG
Smad3	GAGCTTACAAGGCGGCACA	GTTGGGAGACTGGACGAAA
Smad7	TGGTGCGTGGTGGCATACT	CGATCTTGCTCCTCACTTTCTGT
GAPDH	ACAGCAACAGGGTGGTGGAC	TTTGAGGGTGCAGCGAACTT

The article "Sulodexide Prevents Peritoneal Fibrosis by Downregulating the Expression of TGF-β1 and Its Signaling Pathway Molecules" was retracted in 2023. Reasons: signs of a paper mill; compromised peer review; unreliable results or conclusions.

## Data Availability

The data used and analyzed during the current study are available from the corresponding author upon request.
